The article "The Valuable Role of ARMC1 in Invasive Breast Cancer as a Novel Biomarker" was retracted in 2024. Reasons: signs of a paper mill; suspected computer-generated content; unreliable results or conclusions; concerns about the data.

# The Valuable Role of ARMC1 in Invasive Breast Cancer as a Novel Biomarker

**DOI:** 10.1155/2022/1740295

**Published:** 2022-03-26

**Authors:** Yunhao Gan, Fuxin Zhong, Hao Wang, Lingyu Li

**Affiliations:** ^1^Institute of Neuroscience, Department of Pathology, Chongqing Medical University, China; ^2^Institute of Neuroscience, Department of Human Anatomy, Chongqing Medical University, China; ^3^Department of Breast Surgery, People's Hospital of Yubei District of Chongqing, China; ^4^Department of Pathology, Chongqing Medical University, China

## Abstract

**Background:**

Invasive breast carcinoma (BRCA) is a common type of breast cancer with a high clinical incidence. Thus, it is significant to find effective biomarkers for BRCA diagnosis and treatment. Although some members of armadillo (ARM) repeat family of proteins are confirmed to be biomarkers in cancers, the role of armadillo repeat-containing 1 (ARMC1) in BRCA remains unknown.

**Methods:**

We firstly analyzed the ARMC1 expression in normal breast tissues and BRCA samples and its association with overall survival by the public database. Next, the *χ*^2^ test was used to evaluate the prognostic significance of ARMC1 expression in TCGA-BRCA patient samples. The ARMC1 mutations in BRCA were explored in the cBioportal database. Besides, the Gene Ontology (GO) and Kyoto Encyclopedia of Genes and Genomes (KEGG) enrichment analyses were used to explore the biological functions of ARMC1 in BRCA. Finally, immunohistochemistry and immunofluorescence staining were performed to validate the ARMC1 expression in BRCA.

**Results:**

ARMC1 expression in tumor samples was significantly higher than that in normal tissues, and higher expression of ARMC1 was related to lower survival. Moreover, the tumor stage and histology of BRCA patients were associated with ARMC1 expression. ARMC1 genetic mutations occurred in 32% of BRCA patients, and the amplification and high expression of ARMC1 accounted for most of them. Furthermore, functional enrichment analysis suggested that ARMC1 might be involved in the cell cycle in BRCA. Ultimately, increased ARMC1 expression was found in clinical breast carcinoma tissues by our confirmatory experiments.

**Conclusions:**

ARMC1 may play a significant role in BRCA and act as a biomarker, which provides valuable clues for the treatment and diagnosis of BRCA.

## 1. Introduction

Breast cancer is one of the most prevalent female malignancy, and it is also the main cause of cancer death in women [1, 2]. Currently, mammography and magnetic resonance imaging are the primary approaches for diagnosing breast cancer in clinical practice [3]. In terms of treatment, radical mastectomy, radiotherapy, and chemotherapy were the preferred methods for breast cancer [4]. With the improvement of screening ability and detection technology, the diagnosis and therapy for invasive breast carcinoma (BRCA) have made ideal progress in recent years [5]. However, a large number of patients are still diagnosed with BRCA each year, and it is also the second common cause of cancer death in women [6]. Therefore, exploring novel biomarkers remains to be crucial for BRCA.

The article "The Valuable Role of ARMC1 in Invasive Breast Cancer as a Novel Biomarker" was retracted in 2024. Reasons: signs of a paper mill; suspected computer-generated content; unreliable results or conclusions; concerns about the data.

In searching potential biomarkers for BRCA, we discovered that the armadillo (ARM) repeat proteins family is widely involved in cancer progression. Recent researches have revealed that ARM repeat proteins have diverse works in many eukaryotes through their ARM repeat structure [7]. Several ARM repeat proteins have been demonstrated to be involved in tumor development and metastasis. As a famous member of the ARM repeat protein family, *β*-catenin expression in the cytoplasm and nuclear transfer can promote prooncogene transcription such as c-Myc and CyclinD-1 by the Wnt/*β*-catenin signaling pathway [8, 9]. In addition, the interaction between ARMC12 and retinoblastoma binding protein 4 can promote neuroblastoma progression by inhibiting the transcription of tumor suppressor genes [10]. However, some members of ARM repeat protein family can also inhibit the development cancer. For example, adenoma polyposis coli (APC) can degrade the *β*-catenin through glycogen synthase kinase 3*β* (GSK3*β*), thereby blocking Wnt/*β*-catenin cancer signaling in colorectal cancer [11]. Armadillo repeat-containing 1 (ARMC1) was originally found in mitochondrion as a structural subunit [12]. Its coding gene locates at position 8q13.1 of the human chromosome. Similar 42 amino acid repeats define it as a member of the ARM family. However, the role of ARMC1 in BRCA remains unclear, so it is of great significance to study the role of ARMC1 in breast cancer.

This study is aimed at exploring whether ARMC1 acts as a valuable biomarker of BRCA. Therefore, we firstly investigated the expression of ARMC1 and evaluated the prognostic significance of ARMC1 in TCGA-BRCA patients. Moreover, we also explored ARMC1 genetic mutations in BRCA and the role of ARMC1 coexpressed genes in cell cycle regulation. Eventually, we validated the ARMC1 expression level in clinical breast tissues. Thus, this study may contribute to the clinical treatment of BRCA.

## 2. Methods

### 2.1. Gene Expression Profiling Interactive Analysis

The Gene Expression Profiling Interactive Analysis (GEPIA, http://gepia.cancer-pku.cn/) is a web-analysis tool based on TCGA and GTEx data, which provide interactive and customizable functions including differential expression analysis, profiling plotting, correlation analysis, and patient survival analysis [13]. Thus, GEPIA database was used to explore ARMC1 expression and its overall survival in BRCA samples.

The article "The Valuable Role of ARMC1 in Invasive Breast Cancer as a Novel Biomarker" was retracted in 2024. Reasons: signs of a paper mill; suspected computer-generated content; unreliable results or conclusions; concerns about the data.

### 2.2. Kaplan-Meier Plotter

Kaplan-Meier plotter (http://kmplot.com/analysis/) is a widely used online-analysis tool for prognostic value with plentiful gene expression data and relevant clinical data [14]. Kaplan-Meier plotter was performed to analyze the prognostic value of ARMC1 in BRCA.

### 2.3. Human Protein Atlas

Human Protein Atlas (HPA) database (https://www.proteinatlas.org) is a tool for validating immunohistochemistry-based protein expression patterns and extending the map of protein expression patterns in cancer research projects [15]. HPA was used to search the mRNA and protein expression levels of ARMC1 and analyze the prognostic evaluation of ARMC1 in BRCA.

### 2.4. The Cancer Genome Atlas

The Cancer Genome Atlas (TCGA, https://portal.gdc.cancer.gov/) is a public database that provides large cancer genomic profiles of over 30 human tumors; its primary purpose is to research individual cancer types through large-scale genome sequencing and integrated multidimensional analyses [16]. TCGA database was used to collect the BRCA cases with ARMC1 differentially expression for prognostic evaluation and risk factor analysis. The TCGA RNA-seq data and corresponding clinical information of 869 BRCA samples were downloaded from TCGA.

### 2.5. cBio Cancer Genomics Portal

The cBio Cancer Genomics Portal (http://cbioportal.org) is an open-access database, which provides more than 5,000 tumor samples from 20 cancer studies to explore multidimensional cancer genomics data sets [17]. The cBio Cancer Genomics Portal database was used to find the genetic mutations of ARMC1 in BRCA and coexpressed genes associated with ARMC1.

### 2.6. Metascape

Metascape (http://metascape.org/gp/) is a web-based portal that combines works including functional enrichment, interactome analysis, gene annotation, and membership search [18]. Metascape was used to analyze the signaling pathways based on the coexpressed genes related to ARMC1 expression.

### 2.7. DAVID Functional Annotation Tool

DAVID Bioinformatics Resources (DAVID/https://david.ncifcrf.gov/) is a functional annotation tool with public bioinformatics resources. It provides over 40 available annotation categories at the gene and protein level [19]. DAVID was used to perform GO and KEGG analysis based on the coexpressed genes associate with ARMC1.

### 2.8. Patient Selection

According to the situation that ARMC1 is mainly mutated in invasive ductal carcinoma and invasive lobular carcinoma, recent clinically relevant BRCA cases (10 of invasive ductal carcinoma, 5 of invasive lobular carcinoma) that recently appeared in clinical practice were randomly selected. Fifteen pairs of paraffin sections including BRCA tissues and corresponding para-carcinoma tissues were obtained from the Pathological Diagnosis Center of Chongqing Medical University (Chongqing, China). All samples for the confirmatory experiment were selected female patients, and their ages range from 33 to 66 years old. Pathological diagnosis of breast cancer types included invasive ductal carcinoma cases and invasive lobular carcinoma. More characteristics about participants were shown in Supplement Table 1.

The article "The Valuable Role of ARMC1 in Invasive Breast Cancer as a Novel Biomarker" was retracted in 2024. Reasons: signs of a paper mill; suspected computer-generated content; unreliable results or conclusions; concerns about the data.

### 2.9. Cell Line and Their Extraction

Human breast carcinoma cell lines (MCF-7) and human normal breast cells (MCF-10A) were used for in vitro experiments, which were purchased from Procell Life Science&Technology (Wuhan, China). MCF-7 cells were maintained in Dulbecco's Modified Eagle Medium (DMEM; Gibco, Carlsbad, USA) supplemented with 10% fetal bovine serum (FBS) and 10 *μ*/ml penicillin G/streptomycin, and MCF-10A were maintained in 10A cell-specific culture medium (Procell Life Science&Technology). Both cell lines were maintained at 37°C in a humidified atmosphere containing 5% CO2.

Get rid of the culture medium from the petri dish and wash it three times with phosphate-buffered saline (PBS). Cells were collected by scraping off after the addition of cell lysis buffer (Beyotime, Shanghai) and then mixed and place at a standstill for 30 minutes. Collect cell sample by extracting supernatant after centrifugation.

### 2.10. Quantitative Reverse Transcription-Polymerase Chain Reaction (qRT-PCR)

Total RNA of all samples in our experiment was extracted using the M5 Universal RNA Mini Kit (Mei5bio, Beijing). Cells were collected by scraping with phosphate-buffered saline (PBS) and extracting the supernatant after mixing well with 500 *μ*l lysis solution. The supernatant was added with an equal volume of 70% ethanol and transferred to an adsorption column for centrifugation. Add protein solution RW and repeat centrifugation. Next, add rinse solution to the adsorption column and centrifuge (twice). Lastly, add 50 *μ*l RNase-Free H2O to the adsorbed membrane according to the expected RNA yield. The measured RNA concentration is 429 ng/*μ*l (MCF-7) and 459 ng/*μ*l (10A). Then, we conducted reverse transcription assays using the M5 Sprint qPCR RT kit with gDNA remover (Mei5bio, Beijing). The total volume of the cDNA reaction system was 10 *μ*l. The quantitative polymerase chain reaction (q-PCR) analysis was performed using CFX Connect Real-Time System (Bio-Rad, USA). Predenaturation was performed at 95°C for 30 s and cycled once. PCR reaction was performed at 95°C for 5 s and 60°C for 20 s, cycled 40 times. Fusion curve analysis at 95°C for 0 s and 65°C for 15 s. The following primer sequences for this assay were used: armadillo repeat-containing 1 (ARMC1): (forward): 5′-AACTACAAACAAACGTGCCAAAA-3′; (reverse): 5′-ACACACCTTTGAACACACCTATT-3′; glyceraldehyde-3-phosphate dehydrogenase (GAPDH): (forward): 5′-GGACACTGAGCAAGAGAGGC-3′; (reverse): 5′-TTATGGGGGTCTGGGATGGAA-3′. All the primer sequences came from Tsingke Biotechnology (Beijing, China).

The article "The Valuable Role of ARMC1 in Invasive Breast Cancer as a Novel Biomarker" was retracted in 2024. Reasons: signs of a paper mill; suspected computer-generated content; unreliable results or conclusions; concerns about the data.

### 2.11. Enzyme-Linked Immunosorbent Assay

This experiment was completed by using the ARMC1 enzyme-linked immunosorbent assay kit (Jiangsu Jingmei Biological Technology, China). Dilute the standard according to concentration size order, and then incubate the test plate for 30 minutes at 37°C after adding the standard, sample, and distilled water to programmed standard holes, sample holes, and blank. Put the prepared cleaning solution in each hole and shake it for washing the plate, and then tap the plate gently to get rid of the cleaning solution. Repeat this clean step after the addition of the enzyme-labeled reagent except for the blank. The developing color solution was added to each hole and placed statically at 37°C for 15 minutes in the dark. Lastly, read the results after the addition of the stop solution. The Prime 8 software was used to analyze the results of ELISA.

### 2.12. Immunohistochemistry (IHC) Analysis

This experiment was performed by mouse/rabbit streptavidin-biotin assay system (ZSGB-BIO, Beijing). IHC assays were performed using formalin-fixed BRCA tissue samples which were embedded in 4 *μ*m thick paraffin sections. Paraffin sections were deparaffinized by graded alcohol and then incubated by endogenous peroxidase blockers for 20 minutes. The sections were incubated with antibodies against ARMC1 (Novus Biologicals, USA) overnight at 4°C after Goat Serum Blocking Solution incubation. Incubate slides with the secondary antibody for 15 minutes at room temperature, and then incubate the slides with horseradish enzyme-labeled streptavidin for 10 minutes after clearing the secondary antibody. The Image-Pro Plus 6.0 software was used to perform semiquantitative scoring of the images.

### 2.13. Immunofluorescence Staining

Tissue sections were deparaffinized by graded alcohol and then washed three times with phosphate-buffered saline (PBS), permeabilized with 0.4% Triton X-100 for 30 min, and blocked with goat serum working liquid (Wuhan Boster Biological Technology, Wuhan, China) for 2 hours after antigen retrieval. The sections were then incubated overnight with mixed primary antibodies at 4°C, washed in PBS to remove unbound primary antibodies, and incubated with secondary antibodies in the dark at room temperature (RT) for 1 hour. The sections were counterstained with 4′, 6 diamidino-2-phenylindole (Sigma-Aldrich) for 5 minutes and washed with PBS. The primary antibodies included mouse anti-ARMC1 (1 : 50; Novus Biologicals, USA), outer mitochondrial membrane marker-rabbit anti-TOM20 (the outer mitochondrial membrane 20) antibody (1 : 200; Wuhan Proteintech, Wuhan, China), and inner mitochondrial membrane marker-rabbit anti-TIM23 (the inner mitochondrial membrane 23) antibody (1 : 200; Wuhan Proteintech, Wuhan, China). The fluorophore-conjugated secondary antibodies used were goat anti-rabbit Alexa Fluor 488 (1 : 500; Abbkine, Wuhan, China) and goat anti-mouse Alexa Fluor 549 (1 : 500; Abbkine, Wuhan, China). Images were captured by confocal laser scanning microscopy (Nikon A1 + R, Japan). The fluorescence intensity was analyzed by using the ImageJ software.

The article "The Valuable Role of ARMC1 in Invasive Breast Cancer as a Novel Biomarker" was retracted in 2024. Reasons: signs of a paper mill; suspected computer-generated content; unreliable results or conclusions; concerns about the data.

### 2.14. Quantification of Staining Expression

The Image-Pro Plus (Version 6.0.0.260) was used to evaluate the ArmC1 expression in immunohistochemistry. Measure the AOI (area of interest) including average radius, perimeter, and optical density of staining position. After statistics, the IOD (integrated optical density) was calculated by density (mean)∗area density. The expression level was judged from the ratio of SUM value of IOD to SUM value of area.

### 2.15. Statistical Analysis

Receiver operating characteristic (ROC) curve analysis was used to settle the optimal cutoff value of the ARMC1. The optimal cutoff value of the ARMC1 was determined by the maximization of the Youden's index (Sensitivity-(1-Specificity)). Relations of the ARMC1 to other variables were evaluated using the *χ*^2^ test or Spearman's rank correlation coefficient. All statistical analyses were performed using the SPSS version 23.0 software. *p* < 0.05 was considered to indicate a significant difference.

## 3. Result

### 3.1. The Expression Profiles of ARMC1 in BRCA Samples

The expression analysis from the GEPIA database showed that ARMC1 expression in breast tumor samples is higher than that in normal samples (*T* = 1085, *N* = 291) (Figure 1(a)). In addition, a higher ARMC1 expression level was significantly associated with a lower overall survival (*p* < 0.05) (Figure 1(b)). Furthermore, HPA database was used to investigate the mRNA and protein expression of ARMC1 in BRCA. Interestingly, ARMC1 mRNA expression in normal breast tissue was also lower than that in other tissues (Figure 1(c)). On the other hand, we found that ARMC1 mRNA expression in BCRA samples was relatively higher than that in other types of carcinoma (Figure 1(d)). More importantly, ARMC1 protein in breast tissue was significantly higher than that in other tissues (Figures 1(e) and 1(f)).

The article "The Valuable Role of ARMC1 in Invasive Breast Cancer as a Novel Biomarker" was retracted in 2024. Reasons: signs of a paper mill; suspected computer-generated content; unreliable results or conclusions; concerns about the data.

### 3.2. Prognostic Evaluation of ARMC1 Level in BRCA Patients

The Kaplan-Meier plotter tool was used to detect the correlation between ARMC1 expression and overall survival in BRCA. Consistent with the results of GEPIA, high expression of ARMC1 was presented poor prognosis in BRCA (Figure 2(a), hazard ratio (HR) = 1.37, 95% confidence interval (CI):1.23–1.51, *p* = 1.4*E*‐09). In addition, IHC images from the HPA database showed that the intensity and staining in tumor samples were stronger than that in normal samples (Figure 2(b)). Next, the survival analysis in the HPA database confirmed that increased ARMC1 level was associated with poor survival (Figure 2(c)). Furthermore, we explored the risk factors associated with ARMC1 expression in TCGA-BRCA patients. The TCGA-BRCA clinical parameters were collected from the HPA database. Fragments per kilobase per million (FPKM) was used to measure ARMC1 genetic expression. We included 869 patients with seven clinical parameters for this analysis. The average age of the patients was 58 (interquartile range: 48-67). The more specific information of patients is shown in Table 1. The *χ*^2^ test showed that tumor stage (*p* < 0.001), histology (*p* < 0.001), pathological T stage (*p* < 0.001), and pathological N stage (*p* < 0.001) were associated with AMRC1 expression (Supplement Table 2). ROC analysis identified 16.05 as the best cutoff value of ARMC1 by the Youden's index (Sensitivity-(1-Specificity)) (Table 2). Curve area is shown in Supplement Figure 1.

### 3.3. The Genomic Mutations of ARMC1 and Its Biological Pathways in BRCA

The data from the cBioPortal database indicates that ARMC1 mutations occurred in 332 (32%) of 994 samples. Most of them were amplified samples; few of them were mutations of fusion and truncating (Figure 3(a)). As shown in Figure 3(b), breast invasive ductal carcinoma was majorly associated with ARMC1 mutations, which were mainly manifested by high mRNA expression and amplification. Besides, the overall survival of the mutated samples was significantly lower than that of patients without mutation (Figure 3(c); altered group = 322, unaltered group = 672, *p* = 0.0203).

In the neighboring genes related to ARMC1 mutation, TP53 (51.24%), TRPS1 (31.99%), and RAD21 (30.75%) were identified as the top three mutant genes (Figure 3(d)). Next, we used these neighboring genes associated with ARMC1 mutations to analyze the biological networks by the DAVID Functional Annotation Tool (Figure 3(e)). In the cellular component, the endoplasmic reticulum membrane and nucleus were significantly related to ARMC1 mutations, and these mutations affect the activity of various important ion channel modulators including chloride, calcium, and sodium. Mitochondrial permeability regulation and cell death were also identified be involved in these mutations. In biological processes, some vital functions include positive regulation of transporter activity, chromosome organization, sodium ion transportation, homeostasis, and regulating DNA binding transcription factor activity were significantly related to ARMC1 mutations.

The article "The Valuable Role of ARMC1 in Invasive Breast Cancer as a Novel Biomarker" was retracted in 2024. Reasons: signs of a paper mill; suspected computer-generated content; unreliable results or conclusions; concerns about the data.

### 3.4. Enrichment Analysis of Coexpressed Genes Relating to ARMC1 in BRCA

We discover the coexpressed genes positively or negatively associated with ARMC1 in BRCA. As shown in Figure 4(a), most of these genes were positively correlated with ARMC1. Moreover, GO and KEGG GO and KEGG analyses were performed to explore the biological functions of these genes. Interestingly, these genes were mainly related to nucleoplasm, and the protein binding and poly (A) RNA binding were their primary molecular function. More importantly, biological processes involved in these genes included the cell cycle and positive regulation of transcription from RNA polymerase II promoter, etc. (Figures 4(b)–4(d)). Furthermore, the KEGG analysis also showed the potential effect of these genes in the cell cycle (Figure 4(e)).

### 3.5. ARMC1 Was Highly Expressed in Breast Tumor Tissues and Was Mainly Located in the Mitochondrial Membrane

The qRT-PCR assay showed that the ARMC1 mRNA level in MCF-7 cell lines was higher than that in the MCF-10A cell lines (Figure 5(a), *p* < 0.01). For further quantitative analysis of ARMC1 expression, we performed the enzyme-linked immunosorbent assay in two types of cell lines; the results showed that ARMC1 expression in MCF-7 cell lines was higher than in the MCF-10A cell lines (Figure 5(b), *p* < 0.01). Besides, it was obviously found that in the immunohistochemistry that staining intensity and depth of ARMC1 in BRCA tissues were higher than para-carcinoma tissue (Figure 5(c), *p* < 0.01). According to the previous studies that ARMC1 is mainly localized to the mitochondrial, it could be seen in the results of immunofluorescence that ARMC1 in invasive ductal breast carcinoma and lobular breast carcinoma were localized at the both inner mitochondrial membrane and outer mitochondrial membrane (Figures 5(d)–5(e)).

## 4. Discussion

Invasive breast carcinoma (BRCA) is one of the most common diseases in female patients, and various targeted treatments have been applied to BRCA. However, the heterogeneity and wide invasion make BRCA difficult to be cured completely [20]. In our study, we noticed that the expression of ARMC1 was upregulated in BRCA and upregulation of ARMC1 was associated with poor survival. Next, clinical features including tumor stage, histology, pathological T stage, and pathological N stage were found to be related to ARMC1 expression based on the TCGA-BRCA patient cohort. In addition, we found high mutations of ARMC1 in BRCA patients in public databases, as well as associations between ARMC1 and cell proliferation genes by GO and KEGG analyses, suggesting that ARMC1 may be involved in BRCA development. Thus, this study firstly revealed the role of ARMC1 as a novel biomarker in BRCA and provides a regulatory target for the diagnosis and treatment of BRCA.

The article "The Valuable Role of ARMC1 in Invasive Breast Cancer as a Novel Biomarker" was retracted in 2024. Reasons: signs of a paper mill; suspected computer-generated content; unreliable results or conclusions; concerns about the data.

ARM repeat proteins are initially found in drosophila segment polarity protein as multifunctional protein families [21]. The tandem ARM repeat structure composed of 42 repetitive amino acids enables ARM repeat proteins to participate in intracellular signaling and cytoskeletal regulation [22]. Numerous studies have verified the association of the ARM repeat protein family with tumor development [23, 24]. However, the role of ARMC1 in BRCA remains unclear. In this study, we have found that the ARMC1 mRNA expression in tumor samples was higher than that in normal samples. This differential expression highlights the significance of AMRC1 in BRCA. Next, we further explored the prognostic value of ARMC1 in the TCGA-BRCA cohort. Interestingly, the Kaplan-Meier analysis indicated that upregulation of ARMC1 was significantly associated with poor survival, and the same results were verified in TCGA-BRCA cohort. It could be found that factors such as tumor stage and histology were significantly associated with the prognosis of BRCA by *χ*^2^ test of 869 clinical patient information in the TCGA database. Similarly, recent study also found that the higher stage in breast cancer is usually associated with distant metastasis [25]. Thus, the correlation between ARMC1 and stage may be one of the factors inducing metastasis in BRCA.

Numerous analyses of cancer genomes have proven that tumor development is usually accompanied by genetic mutations [26]. The genetic mutations are also recognized as “drivers” for tumorigenesis because of their ability to induce abnormal cell proliferation [27]. Therefore, we attempted to explore the carcinogenesis mechanism of ARMC1 in BRCA from the perspective of gene mutation. The cBio Cancer Genomics Portal database data indicated that 32% of gene mutations were found in BRCA, and amplification and high transcription accounted for most of these mutations. The genetic mutations of ARMC1 were also significantly related to poor survival. Especially, TP53 is one of the highly correlated genes in ARMC1 mutations. The frequent mutations of exon 4 and intron 3 for ARMC1 were reported in breast cancer, which can directly or indirectly cause DNA repair disorders and abnormal cell cycles [28]. Besides, the biological function enrichment showed that ARMC1 and neighboring genes were involved in the positive regulation of transporter activity and regulation of various essential ion channels. It is reported that calcium-activated chloride channels activate EGFR/STAT3 signaling, which can lead to abnormal proliferation of breast cancer cells [29]. Therefore, we speculated that this abnormal ion channel activity caused by ARMC1 mutation may be involved in this signal transduction.

The article "The Valuable Role of ARMC1 in Invasive Breast Cancer as a Novel Biomarker" was retracted in 2024. Reasons: signs of a paper mill; suspected computer-generated content; unreliable results or conclusions; concerns about the data.

Finally, we identified the coexpressed genes associated with ARMC1 and then performed the GO and KEGG analysis of them to explore the regulatory mechanisms of ARMC1 in BRCA. Notably, GO analysis showed that nucleoplasm is majorly associated with ARMC1, and the primary molecular function of them is protein binding. More importantly, KEGG analysis showed that coexpressed genes of ARMC1 were mainly involved in the cell cycle. It has been revealed that cell cycle dysregulation is abnormal cell proliferation [30]. The genes associated with cell cycle regulation such as PRKDC and E2F transcription factor 5 (E2F5) were found in our study. It has been reported that overexpression of PRKDC in breast cancer leads to cell proliferation by accelerating the G2/M cell cycle [31]. In addition, overexpression of E2F5 in breast cancer is also related to cell proliferation [32]. Thus, there are many coexpressed genes associated with ARMC1 that were identified to be involved in cell cycle regulation. ARMC1 may be directly or indirectly involved in breast carcinogenesis by affecting these regulators associated with cell proliferation. However, more studies are required to prove the relationship between ARMC1 and these coexpressed genes in BRCA.

Numerous experiments have found dysregulated ARMC1 in BRCA, which provides concrete evidence that ARMC1 may work as a crucial target in BRCA development and provides a starting point for further study of the ARMC1 mechanism in BRCA. Mitochondria serve as a regulatory center of cellular metabolism; its dysfunction can lead to activation of potential oncogenic pathways [33]. Recently, an increasing number of studies have found that mitochondria can be used as an effective target in breast cancer therapy [34]. It is well-known that mitochondria are an important hub for various ion transport and signal transduction, and ion channels and transporters on mitochondrial bilayer membranes maintain normal cellular homeostasis [35, 36]. There are various ion channels located in the outer or inner mitochondrial membrane that were identified as associated with cancer development. For instance, the overexpression of voltage-dependent anion channels 1 (VDAC1) has been found in cancer cells; it increases the glycolytic rate by the direct mitochondrial ATP transport. This abnormal glucose metabolism promotes the proliferation and migration of tumor cells (the Warburg effect) [37]. Surprisingly, we found that ARMC1 is mainly localized on both the inner and outer mitochondrial membranes in the tissues of the ductal and lobular breast carcinoma. Besides, the ARMC1 mutations may affect various ion channel activities including calcium ions in our result. Thus, ARMC1 may affect BRCA development by mitochondrial ionic homeostasis. Although ARMC1 acts as a molecule on the mitochondrial membrane, the mechanism of ARMC1 in BRCA remains unknown. Therefore, we expect more studies in the future to explore the possible regulatory mechanism of ARMC1 in BRCA through mitochondrial energy metabolism.

The article "The Valuable Role of ARMC1 in Invasive Breast Cancer as a Novel Biomarker" was retracted in 2024. Reasons: signs of a paper mill; suspected computer-generated content; unreliable results or conclusions; concerns about the data.

## 5. Conclusion

Our results suggest that ARMC1 could be a potential biomarker in invasive breast cancer; it provides valuable clues for the treatment and diagnosis of invasive breast cancer. However, this experiment has some limits. Reliable prognostic model analysis cannot be performed due to the limited information of the TCGA-BRCA patient cohort. Thus, more attempts are needed to demonstrate the effect of ARMC1 on the prognosis of BRCA from other pathways.

## Figures and Tables

**Figure 1:** The ARMC1 expression profiles in normal and tumor samples. (a) The ARMC1 expression profile and boxplot in normal samples and BRCA samples. (b) The overall survival associated with ARMC1 expression. (c) The ARMC1 mRNA expression in normal breast tissue. (d) The ARMC1 mRNA expression in tumor samples. (e) The ARMC1 protein expression in normal samples. (f) The ARMC1 protein expression in tumor samples. ARMC1: armadillo repeat-containing 1.

**Figure 2:** ARMC1 expression and prognostic evaluation in BRCA samples. (a) High ARMC1 level was associated with lower survival. (b) Immunohistochemistry images display that ARMC1 expression in tumor tissue was higher than that in the normal tissue. (c) Survival analysis in the HPA database showed increased ARMC1 expression associated with poor survival. HR: hazard ratio; ARMC1: armadillo repeat-containing 1; HPA: Human Protein Atlas.

**Figure 3:** The mutations of ARMC1 in BRCA and its neighboring genes enriched analysis. (a) The genetic mutations of ARMC1 in BRCA. (b) The cancer types with frequent ARMC1 mutations. (c) The overall survival status associated with ARMC1 mutations. (d) Neighborhood gene network diagram of ARMC1 mutations. (e) Biological function analysis of neighboring genes with ARMC1 mutation. ARMC1: armadillo repeat-containing 1; BRCA: invasive breast carcinoma.

The article "The Valuable Role of ARMC1 in Invasive Breast Cancer as a Novel Biomarker" was retracted in 2024. Reasons: signs of a paper mill; suspected computer-generated content; unreliable results or conclusions; concerns about the data.

**Figure 4:** Coexpressed genes with ARMC1 and their enrichment analysis: (a) volcano plot showing coexpressed genes associated with ARMC1; (b) cellular components; (c) biological processes; (d) molecular functions; (e) KEGG pathways. ARMC1: armadillo repeat-containing 1; KEGG: Kyoto Encyclopedia of Genes and Genomes.

**Figure 5:** Validation of ARMC1 expression in BRCA tissues. (a) ARMC1 mRNA level was higher in MCF-7 cell lines compared with MCF-10A (*n* = 10 in each group; ^∗∗∗∗^*p* < 0.0001 versus controls, Student's *t*-test). (b) ARMC1 was higher expressed in MCF-7 cell lines compared with MCF-10A (*n* = 15 in each group; ^∗∗∗∗^*p* < 0.0001 versus controls, Student's *t*-test). C ARMC1 was higher expressed in BRCA tissues than that in para-carcinoma tissues (*n* = 10 in each group; ^∗∗∗^*p* < 0.001 versus controls, Student's *t*-test). Scale bar: 50 *μ*m. (d) ARMC1 was colocalizes with TOM20 in BRCA tissues. (e) ARMC1 was colocalizes with TIM23 in BRCA tissues. Scale bar: 12.5 *μ*m. ARMC1: armadillo repeat-containing 1; BRCA: invasive breast carcinoma; TOM20: the outer mitochondrial membrane 20; TIM23: the inner mitochondrial membrane 23; MCF-7: human breast carcinoma cell lines; MCF-10A: human normal breast cells.

**Table 1:** Clinicopathological characteristics of BRCA samples.

	No. (%)
Location	
Left site	443 (51)
Right site	419 (48.2)
Unknown	7 (0.8)
Histology	
Ductal carcinoma	608 (70)
Lobular carcinoma	215 (24.7)
Other types of carcinoma	45 (5.2)
Unknown	1 (0.1)
Nathologic tumor stage	
Stage I	156 (18)
Stage II	498 (57.3)
Stage III	189 (21.7)
Stage IV	12 (1.4)
Unknown	14 (1.6)
Nodal status	
N+	442 (50.9)
N-	408 (47)
Unknown	19 (2.1)
Nodal status, nr. of +	
0	367 (42.2)
1-3	249 (28.6)
4-9	85 (9.8)
≥10	50 (5.8)
Unknown	118 (13.6)
Lymphovascular invasion	
Present	442 (50.9)
Absent	408 (47)
Unknown	19 (2.1)
T stage	
T1	240 (27.6)
T2	493 (56.7)
T3	98 (11.3)
T4	28 (3.2)
Unknown	10 (1.2)
N stage	
N0	408 (46.9)
N1	296 (34.1)
N2	88 (10.1)
N3	58 (6.7)
Unknown	19 (2.2)

N+: lymph node positive; N-: lymph node negative; BRCA: invasive breast carcinoma.

**Table 2:** The significant ROC curve parameter for the cutoff of ARMC1 expression.

Parameter	AUC	95% CI	Sensitivity	Specificity	Cutoff value	Youden index	*p* value
FPKM	0.803	0.753-0.853	0.761	0.293	16.05	0.467	<0.001

AUC: area under the ROC curve; CI: confidence interval; ROC: receiver operating characteristic curve; ARMC1: armadillo repeat-containing 1. ^∗^Statistically significant (*p* < 0.05).

The article "The Valuable Role of ARMC1 in Invasive Breast Cancer as a Novel Biomarker" was retracted in 2024. Reasons: signs of a paper mill; suspected computer-generated content; unreliable results or conclusions; concerns about the data.

## Data Availability

The data used to support the findings of this study are included within the article.

## Abbreviations

BRCA: Invasive breast carcinoma
ARMC1: Armadillo repeat-containing 1
GO: Gene Ontology
KEGG: Kyoto Encyclopedia of Genes and Genomes
ARMC12: Armadillo repeat-containing 12
APC: Adenoma polyposis coli
GSK3*β*: Glycogen synthase kinase 3*β*
GEPIA: Gene Expression Profiling Interactive Analysis
GTEx: Genotype-tissue expression
HPA: Human Protein Atlas
TCGA: The Cancer Genome Atlas
MCF-7: Human breast carcinoma cell lines
MCF-10A: Human normal breast cells
DMEM: Dulbecco's Modified Eagle Medium
FBS: Fetal bovine serum
PBS: Phosphate-buffered saline
AOI: Area of interest
IOD: Integrated optical density
ELISA: Enzyme-linked immunosorbent assay
IHC: Immunohistochemistry
ROC: Receiver operator characteristic curve
mRNA: Messenger RNA
HR: Hazard ratio
CI: Confidence interval
FPKM: Fragments per kilobase per million
TRPS1: Tricho-rhino-phalangeal syndrome 1
GESA: Gene set enrichment analysis
Arm: Armadillo
EGFR: Epidermal growth factor receptor
STAT3: Signal transducer and activator of transcription 3
PRKDC: Protein kinase DNA-activated, catalytic subunit
E2F5: E2F transcription factor 5
VDAC1: Voltage-dependent anion channels 1
ATP: Adenosine triphosphate
RT: Room temperature.

## Supplementary Materials

Supplementary Materials Supplementary Table 1: clinicopathological characteristics of 15 BRCA patients in validated experiments. Supplementary Table 2: correlation of ARMC1 level with clinicopathological characteristics. Supplementary Figure 1: ROC curve indicating the diagnostic significance of ARMC1.
